The article "Optimal Deep Transfer Learning-Based Human-Centric Biomedical Diagnosis for Acute Lymphoblastic Leukemia Detection" was retracted in 2023. Reasons: signs of a paper mill; suspected computer-generated content; unreliable results or conclusions; concerns about the data.

# Optimal Deep Transfer Learning-Based Human-Centric Biomedical Diagnosis for Acute Lymphoblastic Leukemia Detection

**DOI:** 10.1155/2022/7954111

**Published:** 2022-05-30

**Authors:** Manar Ahmed Hamza, Amani Abdulrahman Albraikan, Jaber S. Alzahrani, Sami Dhahbi, Isra Al-Turaiki, Mesfer Al Duhayyim, Ishfaq Yaseen, Mohamed I. Eldesouki

**Affiliations:** ^1^Department of Computer and Self Development, Preparatory Year Deanship, Prince Sattam Bin Abdulaziz University, AlKharj, Saudi Arabia; ^2^Department of Computer Sciences, College of Computer and Information Sciences, Princess Nourah Bint Abdulrahman University, P.O. Box 84428, Riyadh 11671, Saudi Arabia; ^3^Department of Industrial Engineering, College of Engineering at Alqunfudah, Umm Al-Qura University, Mecca, Saudi Arabia; ^4^Department of Computer Science, College of Science & Art at Mahayil, King Khalid University, Abha, Saudi Arabia; ^5^Department of Information Technology, College of Computer and Information Sciences, King Saud University, P.O. BOX 145111, Riyadh 4545, Saudi Arabia; ^6^Department of Computer Science, College of Sciences and Humanities- Aflaj, Prince Sattam Bin Abdulaziz University, Al-Kharj, Saudi Arabia; ^7^Department of Information System, College of Computer Engineering and Sciences, Prince Sattam Bin Abdulaziz University, AlKharj, Saudi Arabia

## Abstract

Human-centric biomedical diagnosis (HCBD) becomes a hot research topic in the healthcare sector, which assists physicians in the disease diagnosis and decision-making process. Leukemia is a pathology that affects younger people and adults, instigating early death and a number of other symptoms. Computer-aided detection models are found to be useful for reducing the probability of recommending unsuitable treatments and helping physicians in the disease detection process. Besides, the rapid development of deep learning (DL) models assists in the detection and classification of medical-imaging-related problems. Since the training of DL models necessitates massive datasets, transfer learning models can be employed for image feature extraction. In this view, this study develops an optimal deep transfer learning-based human-centric biomedical diagnosis model for acute lymphoblastic detection (ODLHBD-ALLD). The presented ODLHBD-ALLD model mainly intends to detect and classify acute lymphoblastic leukemia using blood smear images. To accomplish this, the ODLHBD-ALLD model involves the Gabor filtering (GF) technique as a noise removal step. In addition, it makes use of a modified fuzzy c-means (MFCM) based segmentation approach for segmenting the images. Besides, the competitive swarm optimization (CSO) algorithm with the EfficientNetB0 model is utilized as a feature extractor. Lastly, the attention-based long-short term memory (ABiLSTM) model is employed for the proper identification of class labels. For investigating the enhanced performance of the ODLHBD-ALLD approach, a wide range of simulations were executed on open access dataset. The comparative analysis reported the betterment of the ODLHBD-ALLD model over the other existing approaches.

## 1. Introduction

For integrating computers closely with experts in the biomedical field, academicians and healthcare professionals are mainly based on human-centric biomedical diagnosis (HCBD) and its fundamental technologies in the biomedical field [1]. The biomedical images attained from various imaging modalities have been classified by the use of conventional statistics using hypothesis testing or Bayesian inference, depending upon regularly disrupted assumptions [2]. A significant solution is to utilize deep learning (DL) models in the knowledge-based system in which the high-dimensional relationship among the datasets is derived. Acute leukemia is an illness related to the kind of blood cancer represented by the irregular propagation of blast cells in the bone marrow that results in replacing the healthy cells and reducing haematopoietic lines in peripheral blood. Quantitative inspection of blood samples plays a vital role in the examination of leukemia [3, 4]. Acute lymphoblastic leukemia (ALL) and acute myeloid leukemia (AML) are two distinct kinds of leukemia, which result in moderate severity when not identified at an earlier stage. AML disturbs the myeloid organ while the ALL can be observed from the bone marrow [5]. ALL is an important haematopoietic illness caused by irregular production of white blood cells (WBCs). Due to the rise in the growth of malignant WBCs, the combat ability of the body with outside materials gets reduced [6]. Till now, the identification of the disease is mainly based on the knowledge and experience of haematologists/pathologists. For supporting the haematologist, computer-aided systems can be employed to categorize the blood cells into normal and affected [7].

Imaging analysis, visual morphological features, and machine learning (ML) techniques are widely adopted to resolve the issues that exist in traditional models. The recent developments of deep learning (DL) have concentrated on the view of classification models by the use of a convolution neural network (CNN) [8]. The utilization of automated classification models can improve the performance of the decision-making process in the biomedical sector [9]. It can be employed for the detection of normal WBCs and the differentiation of particular kinds of cells like erythroid and myeloid precursors. For morphological grouping of cells flowing in peripheral blood, several studies have used CNN models, whereas other models make use of feature extraction and ML based classification models [10].

Numerous CAD models have been available in the literature for acute lymphoblastic leukemia detection. Traditional image processing and machine learning (ML) processes comprised of segmentation, feature extraction, and classification are included. Particularly, segmentation and feature extraction are found to be difficult due to the high variations of the blood smear images attained under diverse condition and significant morphological modifications amongst blast cells. Though few existing models are found to be faster and cost effective compared to manual inspection, the performance and accuracy remain inadequate. Owing to high intraclass variability and interclass resemblance, the subkinds are hard for detection and classification. It becomes necessary to get proper classification as the subclasses act as an important part to assist doctors significantly. After investigating the previous related work, we come to the point that there is still room available for research for the improvement of leukemia detection accuracy.

This study develops optimal deep transfer learning-based human-centric biomedical diagnosis model for acute lymphoblastic leukemia detection (ODLHBD-ALLD). The presented ODLHBD-ALLD model involves the Gabor filtering (GF) technique as a noise removal step with a modified fuzzy c-means (MFCM) based segmentation technique. Moreover, the competitive swarm optimization (CSO) algorithm with the EfficientNetB0 model is utilized as a feature extractor. Furthermore, the attention based long-short term memory (ABiLSTM) model is employed for the proper identification of class labels. In order to assess the improved outcomes of the ODLHBD-ALLD model, a complete experimental analysis is done on the open access dataset. In short, the key contribution of the study is listed below:

  An intelligent CAD model named ODLHBD-ALLD technique for acute lymphoblastic leukemia detection is presented. To the best of our knowledge, the ODLHBD-ALLD model has been never presented in the literature.
  The proposed ODLHBD-ALLD model encompasses GF-based noise elimination, MFCM-based segmentation, EfficientNetB0-based feature extraction, CSO-based hyperparameter optimization, and ABiLSTM-based classification.
  The ODLHBD-ALLD model comprises CSO-based hyperparameter optimization process which helps to boost the classification performance of the proposed model.

## 2. Related Works

This section reviews the recently developed ALL classification models. In reference [11], an unsupervised learning technique such as k-means was employed to segment the nucleus and cytoplasm. Several color and geometric features were removed for analyzing the malignant and healthy leukocyte cells. These features are then exposed to feature removal for reducing the high-dimension feature space to an optimum sized feature set utilizing principal component analysis (PCA). In addition, several binary classification models are utilized to classify the removed regions as cytoplasm, nucleus, and background cells. The authors in reference [12] projected an automated diagnostic model for detecting ALL utilizing a CNN technique. This technique utilizes labeled microscopic blood smear images for detecting malignant leukemia cells. The present work utilizes data attained in the ALL Image Data Base (ALL_IDB) and achieves many data augmentation approaches for increasing the amount of trained data that in effect decreases the over-training problem.

Alsalem et al. [13] presented a structure that supports these departments from estimating, benchmarking, and ranking obtainable multiclass classification (MCC) approaches to the selective of optimum one. This study designed a decision matrix (DM) dependent upon the crossover of 2 groups of multievaluation conditions and 22 MCC methods. Next, the multicriteria decision-making (MCDM) approaches were utilized in the benchmarking and ranking of MCC techniques. Boldú et al. [14] established a DL-based method for predicting the analysis of acute leukemia utilizing blood cell images. For determining an optimum infrastructure for acute leukemia classifier models are estimated. The fine-tuned is executed to these pretrained CNNs for adapting their layers to our data. When the optimum structure is selected, the system with 2 elements working sequentially is configured (ALNet).

Anilkumar et al. [15] purposes for classifying ALL model by DL-based approaches. This analysis utilized DCNN for classifying ALL based on the WHO classifier model without utilizing some image segmentation and feature extraction, which contains intense computation. An image from online image bank of the American Society of Haematology (ASH) is utilized as the classifier. Das et al. [16] projected an effectual and computationally effective ALL recognition approach. It is projected 3 methods by establishing a fully connected (FC) layer and/or dropout layer from the ResNet50 design. In these 3 methods, the model that showcases the optimum trained performance was chosen for extracting features effectually. Finally, it can be executed with SVM, RF, and LR for classifying ALL and relating its performance.

## 3. The Proposed Model

In this article, a novel ODLHBD-ALLD model was developed to notice and categorize acute lymphoblastic leukemia using blood smear images. The proposed ODLHBD-ALLD model involves different stages of subprocesses encompassing GF-based preprocessing, MFCM segmentation, EfficientNetB0 feature extractor, CSO-based hyperparameter optimization, and ABiLSTM classification. The workflow of ODLHBD-ALLD approach is illustrated in Figure 1.

### 3.1. GF-Based Preprocessing

At the initial stage, the preprocessing of the blood smear images is carried out using the GF technique. GF is a bandpass filter that is effectively employed for different machine vision and image processing applications [17]. It reduces the variation among the pixels using the weighted averaging technique to smoothen images. It could not holds edge and texture details of the image. The linear translation‐variant function *f*, which defines the filtering procedure, is given below:

(1) $$\begin{array}{c} f\left(p\right)=\underset{q}{\sum }K_{p,q}\left(Q\right)P_{q}\;, \end{array}$$

where *K*_*p*,*q*_ represents every individual pixel *q* placed at pixel *p* in the filter kernel *K*, and *Q* and *P* are guidance and input images, respectively. For instance, the kernel of the Bilateral Filtering (BF) is defined in the following:

(2) $$\begin{array}{c} K_{p,q}\left(Q\right)=\frac{1}{n}\;\exp\;\left(-\frac{{\left\|p-q\right\|}^{2}}{\sigma_{s}^{2}}\right)\exp\;\left(-\frac{{\left\|P_{p}-Q_{q}\right\|}^{2}}{\sigma_{r}^{2}}\right), \end{array}$$

where *n* is a normalization factor and *σ*_*s*_ and *σ*_*r*_ denote the window size of the neighborhood expansion and the variation in the edge amplitude intensity, respectively. The exponential distribution function is commonly used in equation (2) for computing the impact of various spatial distances using exp (‐ ‖*p* − *q*‖^2^/*σ*_*r*_^2^) , and exp (‐‖*P*_*p*_ − *Q*_*q*_‖^2^/*σ*_*r*_^2^) for labelling the contribution of the pixel intensity range.

### 3.2. Image Segmentation Using MFCM Model

During the image segmentation process, the MFCM model gets executed to segment the preprocessed images. The fuzzy membership utilized by the FCM approach is utilized for assigning pixels to all the categories [18]. Assume *X*={*x*_*i*_, *i*=1,2,…, *N|x*_*i*_ ∈ *R*^*d*^} refers to the *N*‐pixel picture, which is separated into *c* class (cluster), with *x*_*i*_ demonstrating the feature data. This technique is an iterative optimized method, which seeks for minimizing the main function *J*_*m*_, which can be represented as the following equation:

(3) $$\begin{array}{c} J_{m}=\overset{c}{\underset{k=1}{\sum }}\overset{N}{\underset{i=1}{\sum }}u_{ki}^{m}{\left\|x_{i}-v_{k}\right\|}^{2}. \end{array}$$

More, this main function determined in equation (3) is immediately adjusted as follows:

(4) $$\begin{array}{c} J_{m}=\overset{c}{\underset{k=1}{\sum }}\overset{N}{\underset{i=1}{\sum }}u_{ki}^{m}{\left\|x_{i}-v_{k}\right\|}^{2}+\frac{\alpha }{N_{r}}\overset{c}{\underset{k=1}{\sum }}\overset{N}{\underset{i=1}{\sum }}u_{ki}^{m}\overset{m}{\underset{ki}{\sum }}{\left\|x_{i}-v_{k}\right\|}^{2}, \end{array}$$

where *N*_*i*_ refers to the cardinality of a set of neighbors falling inside a local window *x*_*i*_ and *N*_*r*_. Adding the second term in equation (4) makes a spatial restriction, which seeks for maintaining continuity on adjacent pixel values around *x*_*i*_. The main function *J*_*m*_ is minimizing a constraint by utilizing an optimized approach. In medicinal images, neighboring pixel/voxel with comparable feature values are named neighboring pixels or voxel. Its present explanation is as follows:

(5) $$\begin{array}{c} v_{ij}^{'}=\frac{v_{ij}^{y}.s_{ij}^{m}}{\sum_{k=1}^{n}v_{kj}^{y}.s_{kj}^{m}},\\ s_{ij}={\left.\underset{k\epsilon N\left(a_{j}\right)}{\sum }\right)}^{V_{ik}}, \end{array}$$

in which *s*_*ij*_ denotes the spatial function which signifies the probability of pixel or voxel *a*_*j*_ cluster. For approximation to *i*^*th*^ cluster, *N*(*a*_*j*_) represents the square window from the spatial domain, which is centered on a pixel or voxel *a*_*j*_ from the spatial domain and *y*, *m* implies the parameters of windows. The stimulated membership value was enhanced by spatial function, and the remains are protected from clustering.

### 3.3. Feature Extraction

In order to effectually extract the feature vectors, the EfficientNetB0 model is employed. In this study, the EfficientNetB0 baseline approach is employed to receive the input image with the size of 224 × 224 × 3 dimensions [19]. It derives the features through the layers via several convolution (Conv) layers by the use of 3 × 3 receptive field and the mobile inverted bottleneck Conv (MIBConv). The EfficientNetB0 model is applied owing to the stable depth, width, and resolution, which offers highly scalable, precise, and easily deployable model. It performs scaling on every dimension by the predefined collection of scaling coefficients. It exhibits effective outcomes with different versions of 0 to 7, indicating a rise in number of parameters and performance. For optimal adjustment of the hyperparameters involved in the EfficientNetB0 model, the CSO algorithm has been employed to it. The newly presented CSO [20] is demonstrated effectively for large‐scale optimization. During all the iterations, the swarm was arbitrarily separated into 2 groups and pairwise competition is executed amongst the particle in all the groups. After every competition, the winner particle was directly taken from next iteration, but the loser particle is upgraded in its position and velocity by learning from the winner particle:

(6) $$\begin{array}{c} v_{l}^{t+1}=R_{1}^{t}v_{l}^{t}+R_{2}^{t}\left(x_{w}^{t}-x_{l}^{t}\right)+\varphi R_{3}^{t}\left({\bar{x}}^{t}-x_{l}^{t}\right),\\ x_{l}^{t+1}=x_{l}^{t}+v_{l}^{t+1}, \end{array}$$

whereas *t* refers the iteration counter, *R*_1_^*t*^, *R*_2_^*t*^, and *R*_3_^*t*^ are 3 arbitrarily created vectors in [0,1]^*n*^, *x*_*w*_^*t*^ and *x*_*l*_^*t*^ signifies the winner and loser particles respectively, ${\bar{x}}^{t}$ indicates the mean position of existing swarm from the iteration *t*, and ∅ controls the effect of ${\bar{x}}^{t}$. The brief procedure of CSO is summarized in Algorithm 1.

The CSO approach develops an FF for achieving increased classifier action. It defines a positive integer for representing the optimal performance of candidate solutions. During this work, the minimized classifier error rate has been assumed as FF is offered in equation (8)). The best solution is a reduced error rate and poor solution gains an increased error rate.

(7) $$\begin{array}{c} \text{fitness}\left(x_{i}\right)=\text{ClassifierErrorRate}\left(x_{i}\right),\\ =\frac{\text{number of misclassified blood smear images}}{\text{Total number of blood smear images}}*100\;. \end{array}$$

### 3.4. Image Classification

In the final stage, the ABiLSTM model has been utilized for the detection and classification of leukemia. The backward propagating LSTM permits it to attain the preceding data in the sequential information when processing the information. Unlike one‐way LSTM, the Bi‐LSTM enhances a layer of reverse LSTM. The reverse LSTM reverses the information and the hidden state synthesize the forward and reverse data such that cells from the network could attain context data simultaneously [21]. The structure of the BiLSTM model is depicted in Figure 2. The reverse layer LSTM is evaluated correspondingly to forward LSTM, except that the direction is reversed to attain the succeeding time data. It is formulated by the following equations:

(8) $$\begin{array}{c} h_{f}=f\left(w_{f^{1}}x_{t}+w_{f^{2}}h_{t-1}\right),\\ h_{b}=f\left(w_{b1}x_{t}+w_{b2}h_{t+1}\right), \end{array}$$

where *h*_*f*_ denotes the forward LSTM network output and *h*_*b*_ represent the reverse LSTM network output. The last resultant of the hidden layer is

(9) $$\begin{array}{c} y_{i}=g\left(w_{o1}*h_{f}+w_{o2}*h_{b}\right). \end{array}$$

The attention process is one of the probabilistic based weighting models, which is based on the attention of brain [22]. It focuses on particular place and ignores other locations. The presented method rises the performance by highlighting significant factors by allocating distinct probability weights to the input. Thus, the Bi-LSTM allocates the class label. Here, the input sequence value is *x*_1_ to *x*_*k*_, the hidden state value is *h*_1_ to *h*_*k*_, and *a*_*ki*_ denotes the attention weight of hidden state for the present input, which is evaluated by the following equations:

(10) $$\begin{array}{c} a_{ki}=\frac{\text{ exp }\left(e_{ki}\right)}{\sum_{j=i}^{Tx}\text{ exp }\left(e_{kj}\right)},\\ e_{ki}=vTanh\left(Wh_{k}+Uh_{i}+b\right),\\ C=\overset{Tx}{\underset{i=1}{\sum }}a_{ki}h_{i}. \end{array}$$

*h*_*k*_′ denotes the last hidden state value of the last output, evaluated as

(11) $$\begin{array}{c} h_{k}^{\prime }=H\left(C,\;h_{k\prime }x_{k}\right). \end{array}$$

## 4. Performance Validation

In this section, the performance validation of the ODLHBD-ALLD approach is performed using ALL-IDB1 dataset from Kaggle repository [23]. The ALL-IDB1 dataset comprises 108 images with 49 images under abnormal class and remaining 59 images under normal class.  Figure 3 illustrates sample set of images. The results are assessed under 70% of training data and 30% of testing data.

Figure 4 illustrates the confusion matrix generated by the ODLHBD-ALLD model on 70% of training data. The figure reported that the ODLHBD-ALLD model has correctly identified 40 images under normal class and 32 images under abnormal class.

Table 1 and Figure 5 portray the overall classification outcomes of the ODLHBD-ALLD approach on 70% of training data. The experimental values indicated that the ODLHBD-ALLD model has shown effectual classifier results on both class labels. For instance, in normal class, the ODLHBD-ALLD model has offered *accu*_*y*_, *prec*_*n*_, *reca*_*l*_, *spec*_*y*_, and *F*_score_ of 96%, 100%, 93.02%, 100%, and 96.39%. Similarly, on abnormal class, the ODLHBD-ALLD model has provided *accu*_*y*_, *prec*_*n*_, *reca*_*l*_, *spec*_*y*_, and *F*_score_ of 96%, 91.43%, 100%, 93.02%, and 95.52%. Moreover, the ODLHBD-ALLD model has accomplished average *accu*_*y*_, *prec*_*n*_, *reca*_*l*_, *spec*_*y*_, and *F*_score_ of 96%, 95.71%, 96.51%, 96.51%, and 95.95%.

Figure 6 demonstrates the precision-recall curve examination of the ODLHBD-ALLD model on 70% of the training data. The figure indicates that the ODLHBD-ALLD model has obtained maximum precision-recall values on the classification of normal and abnormal class labels.

Figure 7 exemplifies the confusion matrix created by the ODLHBD-ALLD model on 30% of testing data. The figure conveyes that the ODLHBD-ALLD model has properly recognized 15 images under normal class and 17 images under the abnormal class.

Table 2 and Figure 8 represent the overall classification outcomes of the ODLHBD-ALLD system on 30% of testing data. The experimental values designated that the ODLHBD-ALLD model has revealed capable classifier results on both class labels. For instance, in normal class, the ODLHBD-ALLD model has accomplished *accu*_*y*_, *prec*_*n*_, *reca*_*l*_, *spec*_*y*_, and *F*_score_ of 96.97%, 100%, 93.75%, 100%, and 96.77%. In the same way, in abnormal class, the ODLHBD-ALLD model has reached *accu*_*y*_, *prec*_*n*_, *reca*_*l*_, *spec*_*y*_, and *F*_score_ of 96.97%, 94.44%, 100%, 93.75%, and 97.14%. Along with that, the ODLHBD-ALLD model has accomplished average *accu*_*y*_, *prec*_*n*_, *reca*_*l*_, *spec*_*y*_, and *F*_score_ of 96.97%, 97.22%, 96.88%, 96.88%, and 96.96%.

Figure 9 validates the precision-recall curve inspection of the ODLHBD-ALLD model on 30% of testing data. The figure designates that the ODLHBD-ALLD model has gained supreme precision-recall values in the classification of normal and abnormal class labels.

Next, Figure 10 illustrates the training and validation accuracy inspection of the ODLHBD-ALLD technique on the applied dataset. The figure conveyes that the ODLHBD-ALLD model has offered maximum training/validation accuracy in the classification process.

Next, Figure 11 exemplifies the training and validation loss inspection of the ODLHBD-ALLD approach on the applied dataset. The figure reveals that the ODLHBD-ALLD model has offered decreased training/accuracy loss in the classification process of test data.

Table 3 and Figure 12 report a brief comparative study of the ODLHBD-ALLD model with other ML models. The experimental outcome indicated that the k-NN and BPNN models have resulted to lower classification performance. Afterward, the LSVM and RF techniques we tried to accomplish certainly improved classifier results. Along with that, the ADBRF model has reached reasonable performance with *sens*_*y*_, *spec*_*y*_, *F*_score_, *prec*_*n*_, and *accu*_*y*_ of 96.51%, 96.07%, 96.76%, 97.08%, and 96.42%, respectively. However, the ODLHBD-ALLD model has accomplished superior outcomes with *sens*_*y*_, *spec*_*y*_, *F*_score_, *prec*_*n*_, and *accu*_*y*_ of 96.88%, 96.88%, 96.96%, 97.22%, and 96.97%, respectively.

Finally, a brief comparative examination of the ODLHBD-ALLD model with recent approaches [24] is made in Table 4 and Figure 13. The experimental values indicated that the LSVM-DCT model has been able to least *accu*_*y*_ of 90.75%. Followed by, the SVM-P-Morphological + colour + textural model has offered a slightly improved *accu*_*y*_ of 94.14%.

At the same time, the EOC5-morphological + colour + textural, MLP-Shape + Colour, RF-DOST + PCA, SVM-GLRLM, and ADBRF-DOST + PCA + LDA models have accomplished reasonably *accu*_*y*_  of 96.25%, 96.07%, 96.59%, 96.13%, and 95.97%, respectively. However, the ODLHBD-ALLD model has reached superior performance with maximum *accu*_*y*_ of 96.97%. From the aforementioned tables and figures, it can be obvious that the ODLHBD-ALLD technique has the ability to accomplish maximal leukemia detection and classification outcomes over the other methods.

## 5. Conclusion

In this study, a new ODLHBD-ALLD approach was established for the recognition and classification of ALL on blood smear images. The proposed ODLHBD-ALLD model involves different stages of subprocesses, namely GF-based preprocessing, MFCM segmentation, EfficientNetB0 feature extractor, CSO hyperparameter optimization, and ABiLSTM-based classification. In order to assess the improved outcomes of the ODLHBD-ALLD model, a complete experimental analysis is implemented on open access database. The comparative analysis reported the betterment of the ODLHBD-ALLD model over the other existing approaches. Consequently, the ODLHBD-ALLD model can be exploited as an effectual tool for leukemia discovery. In the future, deep instance segmentation approaches can be used to enhance the performance of the ODLHBD-ALLD model. In addition, the ensemble of the pretrained DL models can be employed to improve the classification performance. Moreover, the proposed model can be tested on large-scale datasets in the future.

## Figures and Tables

**Figure 1:** Workflow of the ODLHBD-ALLD model.

**Figure 2:** Structure of BiLSTM model.

**Figure 3:** Sample images. (a) Abnormal and (b) normal.

**Figure 4:** Confusion matrix of the ODLHBD-ALLD model on 70% of training data.

**Figure 5:** Classification performance of the ODLHBD-ALLD model on 70% of the training data.

**Figure 6:** Precision-recall curve of the ODLHBD-ALLD model on 70% of training data.

**Figure 7:** Confusion matrix of the ODLHBD-ALLD model on 30% of testing data.

**Figure 8:** Classifier outcomes of the ODLHBD-ALLD model on 30% of testing data.

**Figure 9:** Precision-recall curve of the ODLHBD-ALLD model on 30% of testing data.

**Figure 10:** Training/validation accuracy of the ODLHBD-ALLD model.

**Figure 11:** Training/validation loss of the ODLHBD-ALLD model.

**Figure 12:** Comparison of the ODLHBD-ALLD model with other ML models.

**Figure 13:** Comparative *accu*_*y*_ of the ODLHBD-ALLD model with recent approaches.

**Algorithm 1:** The CSO algorithm.

**Table 1:** Classifier outcomes of ODLHBD-ALLD model on 70% of training data.

Class labels	Accuracy	Precision	Recall	Specificity	F-score
Normal	96.00	100.00	93.02	100.00	96.39
Abnormal	96.00	91.43	100.00	93.02	95.52
**Average**	**96.00**	**95.71**	**96.51**	**96.51**	**95.95**

**Table 2:** Classifier outcomes of the ODLHBD-ALLD model on 30% of testing data.

Class labels	Accuracy	Precision	Recall	Specificity	F-score
Normal	96.97	100.00	93.75	100.00	96.77
Abnormal	96.97	94.44	100.00	93.75	97.14
Average	96.97	97.22	96.88	96.88	96.96

**Table 3:** Comparative study of the ODLHBD-ALLD model with ML models.

Methods	Sensitivity	Specificity	*F*-score	Precision	Accuracy
k-NN model	93.70	93.96	94.58	95.27	93.57
BPNN model	94.36	96.52	96.10	96.19	94.65
LSVM model	95.49	95.23	95.99	96.94	95.53
RF model	96.47	96.42	95.99	96.39	95.85
ADBRF model	96.51	96.07	96.76	97.08	96.42
ODLHBD-ALLD	96.88	96.88	96.96	97.22	96.97

**Table 4:** Comparative study of ODLHBD-ALLD model with recent approaches.

Methods	Accuracy
SVM-P-morphological + colour + textural	94.14
EOC5-morphological + colour + textural	96.25
MLP-Shape + Colour	96.07
LSVM-DCT	90.75
RF-DOST + PCA	96.59
SVM-GLRLM	96.13
ADBRF-DOST + PCA + LDA	95.97
ODLHBD-ALLD	96.97

## Data Availability

Data sharing is not applicable to this article as no datasets were generated during the current study
